The article "Innate lymphoid cells in neuroinflammation" was published in 2024. Journal: Front Cell Neurosci.

# Innate lymphoid cells in neuroinflammation

**DOI:** 10.3389/fncel.2024.1364485

**Published:** 2024-02-21

**Authors:** Daria Kveštak, Andrea Mihalić, Stipan Jonjić, Ilija Brizić

**Affiliations:** ^1^Center for Proteomics, Faculty of Medicine, University of Rijeka, Rijeka, Croatia; ^2^Department of Biomedical Sciences, Croatian Academy of Sciences and Arts, Rijeka, Croatia

**Keywords:** innate lymphoid cells, microglia, central nervous system, neuroinflammation, central nervous system disorders

## Abstract

Innate lymphoid cells (ILCs) are largely tissue-resident cells that participate in the maintenance of tissue homeostasis and react early to inflammatory events. Mature ILCs are divided into three major groups based on the transcription factors required for their development and function. Under physiological conditions, ILCs are present within the choroid plexus and meninges while the CNS parenchyma is almost devoid of these cells. However, pathological conditions such as autoimmune neuroinflammation and viral infections of the CNS result in the infiltration of ILCs into parenchyma. In this article, we provide an overview of the involvement and function of the ILCs within the CNS during physiological conditions and in infections, autoimmune diseases, neurodegeneration, and injury.

## Introduction

The central nervous system (CNS) is an immunologically specialized tissue that requires exceptional protection and a balanced immune response (Rua and McGavern, 2018; Alves de Lima et al., 2020). The brain was considered to be an “immune-privileged” site for a long time, which refers to evolutionary adaptation developed to tolerate antigen introduction without inducing a robust immune response (Alves de Lima et al., 2020). However, a plethora of studies demonstrated robust immune responses in the CNS in different pathological conditions including infections, autoimmune neuroinflammation, neurodegenerative diseases and CNS injury (Croese et al., 2021). The CNS consists of two major structures, the brain and spinal cord, which are surrounded by protective physical barriers such as meninges, blood-brain barrier (BBB), blood-meningeal barrier, and blood-cerebrospinal fluid (CSF) barrier (Alves de Lima et al., 2020).

The meninges serve as a CNS barrier, but also represent the interface with the periphery and contribute to CNS homeostasis and immune response (Rua and McGavern, 2018). The meninges consist of three layers – dura mater, arachnoid mater, and pia mater. The dura mater is the outermost layer adjacent to the skull, which is highly innervated, vascularized and contains lymphatics (Aspelund et al., 2015; Louveau et al., 2015). The meningeal network of lymphatic vessels is important for tissue fluid homeostasis, macromolecular clearance, and immune cell trafficking in the brain (Aspelund et al., 2015; Louveau et al., 2015, 2017). Meningeal lymphatics absorb brain interstitial fluid via the glymphatic system (Aspelund et al., 2015), the system of perivascular channels formed by astrocytes that mediates clearance of metabolites from the brain parenchyma, but also delivers nutrients and other substances into the brain parenchyma (Iliff et al., 2012; Bohr et al., 2022). Glymphatic system also allows entry of meningeal immune cell-derived factors and cytokines in the brain, resulting in modulation of CNS function (Rustenhoven and Kipnis, 2019). Under healthy conditions, the meninges are populated by different immune cells, including macrophages, dendritic cells (DCs), innate lymphoid cells (ILCs), mast cells, and B and T lymphocytes, with the highest heterogeneity of immune cells within the dura mater (Alves de Lima et al., 2020). Dura contains permeable blood vessels that allow passage of circulating immune cells and supports robust inflammatory response (Balin et al., 1986). Meningeal macrophages are a major immune population in meninges under healthy conditions, which together with perivascular macrophages are sampling the environment (Alves de Lima et al., 2020). Under homeostatic conditions, an antigen produced in the CNS reaches subarachnoid space via CSF flow and drains into meningeal lymphatic vessels where it can be taken up by meningeal antigen-presenting cells (APCs) (Rustenhoven and Kipnis, 2019). In addition to meningeal macrophages and DCs, mast cells can also act as APCs since they can express both major histocompatibility complex, class I (MHC-I) and class II (MHC-II) molecules (Russi et al., 2018). Therefore, meningeal APCs have the potential to exert a profound influence on T-cell priming and effector function. T-cells occupy distinct spatial localization around the dural sinuses, where lymphatic vessels are present. This spatial localization allows T-cells fast and efficient sampling of the CSF, without entering the CNS parenchyma (Rustenhoven and Kipnis, 2019; Ampie and McGavern, 2022). Due to T-cell expression of distinct chemokine receptors, such as C-C motif chemokine receptor 5 (CCR5), C-X-C motif chemokine receptor 3 (CXCR3) and C-X-C motif chemokine receptor 4 (CXCR4), antigen encounter can result in T-cell migration into CNS parenchyma toward chemokine gradient (Bartholomäus et al., 2009; Ma et al., 2021). Furthermore, T-cell-derived cytokines can modulate neuronal activity directly or indirectly, by acting on glial cells (Choi et al., 2016; Filiano et al., 2016). Another important immune cell population that resides in the healthy meninges is B cells (Ampie and McGavern, 2022). They represent around 30% of resident immune cells in the dura and are detected in multiple stages of development. Resident meningeal B cells are localized extravascularly around dural venous sinuses and are relatively immobile (Ampie and McGavern, 2022). Other immune cells also populate meninges, even though at lower numbers.

The choroid plexus (CP) is located within the ventricles of the brain, it contains the blood-CSF barrier, and the ependymal cells within the CP produce the CSF. CP regulates the entrance of immune cells into the brain, as it contains fenestrated vascular endothelial cells without tight junctions between individual cells, allowing direct contact between CSF and systemic circulation (Ampie and McGavern, 2022). Within the CP there is a network of immune, neuronal, and mesenchymal cells that represent an immunologically active barrier and a key part of CNS neuroimmune interaction. The dominant population of immune cells in the CP are specialized populations of macrophages, which together with bone-marrow-derived DCs, can present antigens to T-cells (Cui et al., 2021). A variety of other immune cells, including mast cells, basophils, monocytes, neutrophils, and lymphocytes are also found in the CP.

In contrast to meninges and CP, the CNS parenchyma is devoid of immune cells under healthy conditions. The exception is microglia, the only brain-resident immune cells and thus the first responders to changes within the CNS parenchyma (Rock et al., 2004; Goldmann et al., 2016). Microglia play an important role during brain development, participating in phagocytosis of synapses during development and secreting growth factors necessary for neuronal survival (Lehnardt, 2010; Paolicelli et al., 2011; Miyamoto et al., 2016; Tsai et al., 2016; Prinz et al., 2021). Changes in tissue microenvironment such as injury, neurodegeneration, or infection of the CNS, can initiate a robust inflammatory response characterized by the activation of microglia and recruitment of peripheral immune cells. Activation of microglia leads to the alteration of their transcriptional profile, expression of various surface markers and the production of pro-inflammatory cytokines and chemokines (Norris and Kipnis, 2019). Astrocytes, like microglia, are activated in response to inflammatory stimuli, which can lead to loss of their ability to maintain the BBB. Peripheral immune cells that infiltrate the brain can further regulate the recruitment of other cells via cytokine secretion (Passaro et al., 2021). The early cellular immune response is characterized by the infiltration of innate immune cells such as macrophages, neutrophils, and natural killer cells (NK cells), followed by the infiltration of adaptive T and B cells into the CNS. Different subsets of T-cells provide help to other immune cells, have important immunoregulatory functions, or recognize and destroy damaged cells (Smolders et al., 2018; Passaro et al., 2021). Upon clearance of the pathogen, T-cells can be retained in the CNS as tissue-resident memory cells to prevent re-infections and dampen inflammatory responses upon reinfection (Wakim et al., 2010; Brizic et al., 2018). Although activation of the immune cells within the brain parenchyma is necessary for the resolution of infections, balanced control of immune response is needed to prevent neuropathology.

## Innate lymphoid cells in the CNS

Innate lymphoid cells are lymphocytes that lack rearranged antigen receptors expressed on T-cells and B-cells, but their transcriptional programs and cytokine secretion mirror those of the different T-cell subsets (Artis and Spits, 2015). Mature ILCs are divided into three major groups based on the transcription factors required for their development, function, and cytokine secretion profiles (Vivier et al., 2018). ILCs are largely tissue-resident cells that contribute to the maintenance of tissue homeostasis and react early to inflammatory events. Although ILCs, except for NK cells, have been described as dominantly tissue-resident cells, data suggests that a proportion of the ILCs can be migratory (Gasteiger et al., 2015; Dutton et al., 2019). For example, both ILC1 and ILC2 populations found in lymph nodes can be tissue-resident but also enter circulation (Dutton et al., 2019). In addition, ILC3 can infiltrate the CNS from the circulation (Grigg et al., 2021). The exact mechanisms driving the recruitment of ILCs into the brain are still not well understood. Due to the existence of brain barriers, ILCs have limited presence under the steady state in the brain parenchyma, however, they are present in significant numbers in the CP and meninges (Figure 1).

**FIGURE 1:** Innate lymphoid cells in the CNS. Under physiological conditions, ILCs are present within the choroid plexus (CP) and meninges while the CNS parenchyma is almost devoid of ILCs. Meninges have more ILC2s relative to ILC3s (Gadani et al., 2017), NK cells and ILC1s (Romero-Suarez et al., 2019). ILC1s are found in the CP, and very few NK cells (Romero-Suarez et al., 2019) and ILC3s (Fung et al., 2020) are present. ILC2s are absent in the CP of young mice, but they accumulate and become dominant population during aging (Fung et al., 2020). Created with BioRender.com.

Group 1 innate lymphoid cells comprise type 1 ILC cells (ILC1s) and NK cells (Vivier et al., 2018). While NK cells develop from a common innate lymphoid progenitor (CILP) via an NK cell precursor, ILC1s develop from CILPs via an innate lymphoid cell precursor. Although ILC1s and NK cells have different developmental paths, both of these cell types produce interferon-gamma (IFN-γ) as their principal cytokine, and are dependent on the transcription factor T-box expressed in T-cells (T-bet), which is required for ILC1 development and terminal maturation of NK cells (Zhang et al., 2018). In contrast to ILC1s, NK cells require the transcription factor Eomesodermin (Eomes) for their development and are cytotoxic (Gordon et al., 2012; Daussy et al., 2014). Even though ILC1s are not cytotoxic in general, liver embryonically derived ILC1s give rise to a cytotoxic subset (Sparano et al., 2022). In addition, ILC1s produce more proinflammatory cytokine tumor necrosis factor alpha (TNF-α) than NK cells in naïve mice (Romero-Suarez et al., 2019). ILC1s have many phenotypic markers in common with NK cells. In mice, both cell types are defined as CD45-positive, CD3-negative, and CD19-negative cells that express NKp46/NK1.1. A particular expression pattern of integrins can be used to differentiate between these two ILC types. While NK cells express the integrin CD49b, ILC1s express the integrin CD49a (Daussy et al., 2014). Since the expression of CD49a is often lost upon cell activation, other more stable markers such as CD200R are used to distinguish ILC1s from NK cells in mice (Weizman et al., 2017). However, approaches for discrimination and characterization of ILC subsets are ever-evolving, especially in the context of different tissues and pathophysiological conditions. Within the naïve CNS, both NK cells and ILC1s are present in the meninges, ILC1s are enriched in the CP where very few NK cells are present, while CNS parenchyma is devoid of these cells under physiological conditions (Romero-Suarez et al., 2019). The physiological functions of NK cells and ILC1s found in the CNS are still not well understood. A recent study has shown that meningeal NK cells and ILC1s can regulate the behavior of mice (Garofalo et al., 2023). Namely, NK cells and ILC1s produce IFN-γ and acetylcholine that shape synaptic neuronal transmission and modulate brain homeostatic functions. Thus, group 1 ILCs seem to establish important functional interactions with neurons under physiological conditions.

Group 2 ILCs consists of a single subset, ILC2s, which produce type 2 cytokines, predominantly interleukin- (IL-) 5 and IL-13, and are defined by the expression of transcription factors GATA binding protein 3 (GATA3) and RAR-related orphan receptor alpha (RORα), required for ILC2 differentiation and maintenance (Vivier et al., 2018). ILC2s are most abundant at mucosal barriers where they act as key initiators of type 2 inflammation and tissue repair and are activated by host-derived cytokines and alarmins. In the naïve CNS, ILC2s reside within the dura meninges of both young (2–3 months old) and aged mice (18–20 months old) (Fung et al., 2020). In the CP of young mice ILC2s are absent, but they accumulate in the CP of aged mice. Almost no ILC2s were labeled with intravenously injected anti-CD45.2 antibody, demonstrating that under physiological conditions ILC2s are non-circulating, brain resident cells. Leptomeninges and brain parenchyma regions, including the cortex, prefrontal cortex, striatum, thalamus, hippocampus, and subventricular zone are devoid of ILC2s (Fung et al., 2020). In mice, meningeal ILC2s express c-kit, IL-33 receptor ST2, CD25 and IL-7Rα and are thus similar to their peripheral counterparts. However, meningeal ILC2s transcriptional profile differs when compared to lung ILC2s, with most of the differentially expressed genes in lung-derived ILC2s being upregulated compared to meningeal ILC2s (Gadani et al., 2017). The enriched gene sets include those relating to inflammation, signal transduction, and metabolism, suggesting an increased basal activation state in the lung relative to meningeal ILC2s (Gadani et al., 2017). Although the basis for the difference between lung and meningeal ILC2s is unclear, lung ILC2s are exposed to far more environmental stimuli than meningeal ILC2s, likely leading to these transcriptional differences. A recent study reported that during development, meningeal ILC2s are required for cortical inhibitory synapse maturation and adult social behavior (Barron et al., 2023). This function of ILC2 seems to be dependent on IL-13-production. Thus, ILC2s have an important role in shaping brain function.

Group 3 ILCs include NK cell receptor positive (NCR^+^), NK cell receptor negative (NCR^–^) ILC3s and the lymphoid tissue inducer (LTi) cells, all of which are dependent on the transcription factor RAR-related orphan receptor gamma (RORγt) and can produce IL-17 and/or IL-22 (Vivier et al., 2018; Fiancette et al., 2021). ILC3s are most abundant at mucosal sites where they play an important role in the regulation of commensal microbiota and provide protection against extracellular bacteria (Vivier et al., 2018; Panda and Colonna, 2019). Different subsets of RORγt^+^ ILC3s corresponding to LTi, NCR^+^ and NCR^–^ ILC3 populations populate the meninges (Hatfield and Brown, 2015; Gadani et al., 2017). Interestingly, the meninges have more ILC2s than ILC3s in the healthy state, and both populations were more numerous in the brain than in the spinal cord meninges (Gadani et al., 2017). In addition to their presence in the meninges, ILC3s are also found in the CP of aged mice (Fung et al., 2020). Functions of this ILC3 subsets in the CNS under homeostatic conditions are ill-defined.

## ILCs in CNS disorders

Pathological conditions such as cerebral ischemia, autoimmune neuroinflammation and viral infections of the CNS result in the infiltration of ILCs into parenchyma (Trifilo et al., 2004; Alsharifi et al., 2006; Thapa et al., 2008; Gan et al., 2014; Hatfield and Brown, 2015; Romero-Suarez et al., 2019; Kveštak et al., 2021; Zheng et al., 2023). The exact role of ILCs within the CNS upon different pathological conditions remains largely unknown. ILCs, and especially NK cells, are also involved in brain cancers. The protective role of NK cells against gliomas is well recognized, and therapeutic approaches exploiting this knowledge are being rapidly developed. However, these aspects of ILC biology are well-covered elsewhere (Sedgwick et al., 2020; Liu et al., 2021; Balatsoukas et al., 2022), and therefore were not covered by this review.

## ILCs and infection

Involvement of group 1 and group 3 ILC subsets in viral infections within the CNS was the subject of several studies (Trifilo et al., 2004; Alsharifi et al., 2006; Thapa et al., 2008; Kveštak et al., 2021; Lee et al., 2022; Martin and Griffin, 2022). Due to the expression of different chemokine receptors, such as CXCR3, CX3C-chemokine receptor 1 (CX3CR1), and CC-chemokine receptor 2 (CCR2), these cells can respond to a large array of chemokines, and can be recruited to the site of inflammation (Trifilo et al., 2004; Thapa et al., 2008; Kveštak et al., 2021). The involvement of ILCs in viral infections of CNS is summarized in Figures 2A–C.

**FIGURE 2:** ILCs in the infections. **(A)** Perinatal MCMV infection leads to infiltration of NK/ILC1 cells into the brain. Both NK cells and ILC1s produce IFN-γ leading to activation of microglia and affect development of the cerebellum (Kveštak et al., 2021). **(B)** Infection with MHV leads to the accumulation of NK cells in the brain, which reduce viral titer by producing IFN-γ (Trifilo et al., 2004). **(C)** Virulent Semliki Forest virus (vSFV) infection causes NK cell infiltration into the CNS where they mediate immunopathology (Alsharifi et al., 2006). **(D)** Infection with *Toxoplasma gondii* (*T. gondii)* leads to the accumulation of both NK cells and ILC1s in the brain, but only ILC1s contribute to control of cerebral *T. gondii* infection via IFN-γ (Steffen et al., 2022). Created with BioRender.com.

Human cytomegalovirus (HCMV) is a double-stranded DNA beta-herpesvirus and the most common causative agent of congenital viral infections in humans that may lead to long-term CNS abnormalities (Boppana et al., 2013). We have shown in a mouse model of congenital CMV infection that NKp46^+^ NK and ILC1 cells infiltrate into the brain, coinciding with the detection of the mouse cytomegalovirus (MCMV) in the tissue (Kveštak et al., 2021). In contrast to adult mice in which NK cells provide key protection against MCMV infection, they are unable to control infection in early life (Rozmanic et al., 2023). Microglial expression of chemokine coding genes *Cxcl9* and *Cxcl10* was upregulated following perinatal CMV infection indicating that the early expression of *Cxcl9* and *Cxcl10* could mediate the recruitment of NK and ILC1 cells into the brain (Kveštak et al., 2021). Accordingly, the blockade of chemokine receptor CXCR3 significantly reduced number of brain-infiltrating NK and ILC1 cells in MCMV-infected mice, emphasizing the importance of CXCR3 receptor in their recruitment. Brain infiltrating NK and ILC1 cells were highly activated, as they expressed markers of activation KLRG1 and CD69. Approximately 40% of NKp46^+^ cells that infiltrated MCMV-infected brains expressed a marker of ILC1 cells, CD200R, while the NK cell signature transcription factor Eomes was expressed in ∼40% of NKp46^+^ cells. Although NK and ILC1 cells were unable to control virus infection in the brain of newborn mice, they orchestrated pathological inflammatory responses. Namely, both NK cells and ILC1 cells produced IFN-γ following MCMV infection leading to impaired development of the cerebellum (Figure 2A). This finding is in agreement with a study showing the presence of NKp46^+^ cells in severe cases of HCMV-infected fetal brains (Sellier et al., 2020), demonstrating an association between fetal brain damage and high levels of NK cells. In addition to their pathogenic role in the CNS, group 1 ILCs also mediate activation of microglia and therefore enhance neuroinflammatory response during MCMV infection (Kveštak et al., 2021). Blockade of IFN-γ abrogated microglial activation and normalized cerebellar development indicating that modulation of the inflammatory response can limit CNS disease caused by MCMV infection. NK cells are recruited into the CNS during infection with other viruses as well, including infection with herpes simplex virus type 2 (HSV-2), mouse hepatitis virus (MHV), Zika virus and virulent Semliki Forest virus (vSFV) (Trifilo et al., 2004; Alsharifi et al., 2006; Thapa et al., 2008; Lee et al., 2022). In the case of MHV, an RNA coronavirus that can cause encephalitis in mice, and Zika virus, an RNA flavivirus that can cause a variety of congenital brain abnormalities, NK cells have an important role in virus control (Trifilo et al., 2004; Lee et al., 2022). Control of MHV infection is dependent on NK cell-derived cytokine IFN-γ and control of Zika virus infection is dependent on NK cell cytotoxicity that requires leukocyte immunoglobulin like receptor B4/glycoprotein 49B (LILRB4/gp49B). A beneficial role in controlling infection by NK cells was associated with protection against meningoencephalitis during Zika virus infection (Lee et al., 2022). However, in the case of vSFV, an RNA alphavirus that causes lethal encephalitis in rodents, the depletion of NK cells significantly extended the survival of mice (Alsharifi et al., 2006). Therefore, NK and ILC1 engagement in virus-infected CNS can result in both adverse and beneficial outcomes.

ILC3s were also found to be important during viral encephalitis. Infection of IL-10-deficient mice with a neuroadapted strain of Sindbis virus (SINV), an RNA alphavirus that can induce encephalomyelitis in mice, resulted in increased production of cytokine transforming growth factor, beta 1 (TGFβ1) by ILC3s (Martin and Griffin, 2022). Enhanced TGFβ1 induction in the absence of IL-10 contributed to the development of T helper (Th)17 responses that resulted in worse clinical outcomes (Martin and Griffin, 2022). Thus, dysregulated ILC3 response during viral infections can be an important contributor to immunopathology.

Beside viruses, ILC subsets are engaged in the immune responses to parasites in the CNS (Figure 2D). Infection with *Toxoplasma gondii (T. gondii)*, a parasite that can infect the brain and trigger neuroinflammation, elicits activation of peripheral NK cells and ILC1s (Klose et al., 2014; Ivanova et al., 2020). Accumulation of both NK cells and ILC1s was observed in the cerebral parenchyma, the CP, and the meninges. By using mice that have diminished numbers of NK cells or ILC1s, it was demonstrated that only ILC1s contribute to the early control of cerebral *T. gondii* infection (Steffen et al., 2022). ILC1s serve as an early source of antiparasitic cytokines IFN-γ and TNF-α, thereby initiating a neuroinflammatory response and restricting cerebral *T. gondii* infection (Steffen et al., 2022). While ILC1 cells contribute to the early control of infection, NK cells were detrimental to the control of chronic *T. gondii* infection (Ivanova et al., 2020). Namely, NK cells were negatively affecting CD8 T-cell response. Accordingly, NK cell depletion augmented CD8 T-cell response and reduced cyst burden in the brain and overall mortality, demonstrating that targeting of NK cells could be used as a therapeutic option (Ivanova et al., 2020). Infection with another parasite, *Angiostrongylus cantonensis*, also results in infiltration of NK cells in the CNS that is dependent on CX3CL1 production, presumably by neurons (Zhang et al., 2021). However, NK cells did not provide protection against parasite, but instead, they aggravated brain damage. Besides NK cells and ILC1s, ILC2s are also engaged in the immune responses to parasites. Interestingly, Cardoso et al. have shown that mucosal neurons regulate type 2 inflammatory response by releasing neuromedin U (NMU), a neuropeptide that directly activates ILC2s in response to parasite *Nippostrongylus brasiliensis* (Cardoso et al., 2017). ILC2s activated with NMU produced innate inflammatory and tissue repair cytokines IL-5 and IL-13, which were important for the control of worm infection, demonstrating that ILC2-neuron interactions can provide tissue protection (Cardoso et al., 2017). The description of neuron-ILCs units in the peripheral organs (Cardoso et al., 2017), raises the question of whether ILCs could also directly communicate with neurons and glial cells within the CNS.

## ILCs in autoimmune neuroinflammation, neurodegenerative diseases, CNS injury, and aging

Innate lymphoid cells have been well studied in the context of neurodegenerative diseases, ischemic disease, aging and autoimmune neuroinflammation (Figure 3).

**FIGURE 3:** ILCs in neurodegenerative diseases, ischemic disease, aging and autoimmune neuroinflammation. **(A)** NK cells are involved in the pathogenesis of Alzheimer’s disease (AD) and amyotrophic lateral sclerosis (ALS). In the AD mouse model, NK cells exacerbate cognitive decline and promote neuroinflammation (Zhang et al., 2020). In the mouse model of ALS, NK cells have a key role in microglial activation (Garofalo et al., 2020). **(B)** In a mouse model of cerebral ischemia NK cells are recruited into the brain in CX3CR1-dependent manner and exert IFN-γ-dependent cytotoxicity on ischemic neurons leading to lesion development (Gan et al., 2014). **(C)** During aging, IL-33 can activate choroid plexus ILC2s, which alleviate aging-associated cognitive decline (Fung et al., 2020). **(D)** Upon EAE induction, upregulation of MHC-II on ILC3s promotes pathological CD4 + T-cell responses in the CNS during autoimmune neuroinflammation (Grigg et al., 2021). Created with BioRender.com.

### Group 1 ILCs

The involvement of ILCs has been demonstrated in the pathogenesis of multiple sclerosis (MS), mostly by using experimental autoimmune encephalomyelitis (EAE), a model of MS (Sadeghi Hassanabadi et al., 2022). EAE is induced in mice by active immunization with myelin antigens mixed with adjuvant (Miller et al., 2010). Immunized mice develop paralysis with infiltration of myelin-specific CD4^+^ T-cells in the white matter of the spinal cord, with myelin-specific CD4^+^ T-cells contributing to disease pathogenesis in this mouse model (Kwong et al., 2017; Milovanovic et al., 2017; Grigg et al., 2021). During the development of EAE, NKp46^+^ ILCs, which include ILC1s and the NKp46^+^ subset of ILC3s, have a pathogenic role (Kwong et al., 2017). Specifically, T-bet-dependent NKp46^+^ ILCs control the onset of IL-17-producing CD4^+^ T-mediated neuroinflammation by generating a proinflammatory-cytokine microenvironment in the meninges, which is necessary for the optimal reactivation and maintenance of Th17 cells in the CNS tissue. In addition, NKp46^+^ ILCs also induce the expression of matrix metalloproteinases and chemokines that facilitate the migration of CD4^+^ T-cells out of meninges into the CNS parenchyma (Kwong et al., 2017). Although NK cells were a numerically dominant NKp46^+^ ILC population, they did not have a major role in Th17-induced neuroinflammation (Kwong et al., 2017). However, in another study, it was shown that acetylcholine-producing NK cells could reduce the intensity of inflammation and autoimmune responses in the brain and spinal cord and reduce brain damage (Jiang et al., 2017). Accordingly, upregulation of cholinergic activity was also observed in peripheral CD56^bright^ NK cells of MS patients and CD56^bright^ NK cells were shown to accumulate in the periventricular brain regions in patients with MS (Rodriguez-Lorenzo et al., 2022). It is well-established that microbiota can affect the production of IFN-γ by NK cells (Ganal et al., 2012). In the case of EAE, the gut microbiome modulated IFN-γ production by meningeal NK cells, which was shown to be essential to maintain a subset of anti-inflammatory astrocytes (Sanmarco et al., 2021). This anti-inflammatory astrocyte subset limited EAE development, thus pointing to the importance of microbiota stimulation of NK cells in the context of EAE. These observations have implications for animal studies in general, as microbiota could potentially explain the discrepancies between different studies. Altogether, group 1 ILCs are important orchestrators of autoimmune responses in the CNS.

In addition to autoimmune neuroinflammation, group 1 ILCs are involved in the pathogenesis of neurodegenerative diseases such as Alzheimer’s disease (AD) and amyotrophic lateral sclerosis (ALS) (Garofalo et al., 2020; Zhang et al., 2020). NK cells are found in the CSF of AD patients (Gate et al., 2020). In a triple-transgenic AD mouse model harboring amyloid β precursor protein (APP_*Swe*_), presenilin 1 (PS1_*M*146*V*_), and microtubule-associated protein tau (Tau_*P*301*L*_) transgenes, NK cells had a striking role in exacerbating cognitive decline and promoting neuroinflammation (Zhang et al., 2020). Furthermore, depletion of NK cells enhanced neurogenesis, reduced microglial proliferative response, and decreased expression of multiple proinflammatory cytokines in microglia. In the mouse model of ALS, NK cells directly kill spinal cord motor neurons in an NKG2D-dependent manner and have a key role in microglial activation (Garofalo et al., 2020). Depletion of NK cells delayed motor impairment and increased survival, and reduced the expression of proinflammatory genes, with the simultaneous increase in expression of the anti-inflammatory markers *chil3*, *arg-1*, and *tgf*β, and ROS scavenger *msod1*, as well as the modulation of other genes associated with a homeostatic neuroprotective microglial phenotype (Garofalo et al., 2020). Moreover, NK cells are found in postmortem sporadic ALS motor cortex and spinal cord, while NKG2D ligands are expressed on postmortem sporadic ALS motor neurons, suggesting a key role of NK cells in onset of ALS and motor neuron loss. Furthermore, NK cells are found in the brains of mice and humans with synucleinopathies, neurodegenerative diseases including Lewy body dementia and Parkinson’s disease (Earls et al., 2020). The accumulation of NK cells in the brain was beneficial in a mouse model of synucleinopathies as depletion of NK cells exacerbated motor symptoms and synuclein (syn) pathology (Earls et al., 2020). Although NK cells are not professional phagocytic cells, human NK cell line NK92 and primary human NK cells from healthy individuals can efficiently internalize and degrade α-syn aggregates via the endosomal/lysosomal pathway (Earls et al., 2020). Thus, NK cells could be able to scavenge extracellular α-syn and could be critical for regulating synuclein pathology. NK cells could exert protection also by producing IFN-γ, cytokine required for activation of microglia which are involved in resolving extracellular α-syn. However, whether NK cells use additional mechanisms to exert protective or detrimental effects in synucleinopathies, AD and ALS remain to be elucidated.

Susceptibility to neurological diseases increases during aging (Hou et al., 2019). NK cells are found to be involved in shaping the neurogenesis potential during aging by negatively impacting neuroblast survival (Jin et al., 2021). Namely, activated NK cells locally proliferate and accumulate in the dentate gyrus of normal aged human and mouse brains. Neuroblasts within the aged dentate gyrus had senescent phenotype and reinforced NK cell activation in an IL-27-dependent manner (Jin et al., 2021). Intriguingly, aged neuroblasts had increased expression of NKG2D ligand RAE1, and NK cells eliminated aged neuroblasts in RAE1-dependent manner *in vitro* (Jin et al., 2021). Accordingly, depletion of NK cells led to sustained improvements in neurogenesis and cognitive function during normal aging. Involvement of other factors induced during aging in dentate gyrus, such as IL-2 and C-C motif chemokine ligand 3 (CCL3) (Jin et al., 2021), that are known to influence NK cell expansion and trafficking (Shi et al., 2011), remains to be determined.

In the case of ischemic disease, NK cells have been reported to have both beneficial and detrimental roles (Gan et al., 2014; Zhang et al., 2014; Wang et al., 2023). NK cells accumulate in brain infarction in both humans and mice (Gan et al., 2014; Zhang et al., 2014). In a mouse model of cerebral ischemia NK cells have a pathogenic role and lead to neuronal death, ischemic brain lesions, and to the neurological deficit typical of stroke (Gan et al., 2014). Ischemic neuron-derived fractalkine recruits NK cells into the brain, where they exert cytotoxicity on ischemic neurons and produce IFN-γ that is key for boosting local inflammation and contributes to lesion development (Gan et al., 2014). In another study, the CXCL10-CXCR3 axis contributed to NK cell accumulation in ischemic brain tissue, and NK cells were found to promote the necrosis of neural cells via IFN-γ (Zhang et al., 2014). In contrast, NK cells had a protective role following the induction of photothrombotic ischemia (Wang et al., 2023). ILC1s, ILC2s and ILC3s were also located within the lesion, but the highest influx was observed for NK cells and ILC1s. C-X-C motif chemokine ligand 12 (CXCL12) expression at the BBB was needed for the recruitment of NK cells toward the lesion in a CXCR4-dependent manner. Importantly, NK cells alleviated neurological deficits of mice as observed by beam-walk sensorimotor test (Wang et al., 2023). The underlying cause for the different roles of NK cells in between the studies is not currently clear. However, different models were used, characterized with different kinetics of NK cells which could potentially explain the discrepancies (Gan et al., 2014; Zhang et al., 2014; Wang et al., 2023). Interestingly, NK cells contribute to the clearance of injured sensory axons in peripheral nerves. Injured sensory axons upregulate the expression of ligands for NK cell activating receptor NKG2D, allowing NK cells to selectively degenerate damaged axons aiding functional regeneration (Davies et al., 2019). Whether such mechanisms operate in the CNS remains elusive.

### Group 2 ILCs

Group 2 ILC functions in the CNS were investigated in the context of aging, CNS injury, and CNS demyelination (Gadani et al., 2017; Fung et al., 2020; Hirose et al., 2020). ILC2s are a major lymphocyte subset in the aged (18–22 months old mice) CP, accounting for up to 50% of the lymphocytes present (Fung et al., 2020). This corresponds to a three- to fivefold increase in ILC2 number in the CP of aged mice as compared to 2–3 months old mice. ILC2s also accumulate in the meninges of aged mice, even though more moderately (Fung et al., 2020). Other ILC subsets, including NK cells, ILC1s, and ILC3s, are barely detectable in the CP of aged mice. In humans, ILC2s are also a major subset of lymphocytes in the CP of aged individuals (Fung et al., 2020). CP ILC2s in the aged mouse brain are long-lived, relatively resistant to cellular senescence and exhaustion, and can switch between cell cycle dormancy and proliferation (Fung et al., 2020). They are functionally quiescent at homeostasis but can be activated by IL-33 to produce large amounts of type 2 cytokines IL-13 and IL-5. Moreover, CP ILC2s possess a more potent ability to proliferate and produce type 2 cytokines than meningeal ILC2s (Fung et al., 2020). Treatment of aged mice with IL-33 leads to the activation of CP ILC2s and alleviates aging-associated cognitive decline, and similarly treatment with IL-5 or adoptive transfer of activated ILC2s drastically enhances cognitive function and spatial memory of aged mice (Fung et al., 2020). Interestingly, the numbers of ILC2s are greatly reduced in aged brain in 7-month-old triple-transgenic AD mice, compared to those in control wild-type mice (Fung et al., 2021). The remaining ILC2s failed to efficiently produce cytokine IL-5 but gained the capability to express a number of proinflammatory genes indicating that group 2 ILCs are numerically and functionally deficient in the triple transgenic mouse model of AD (Fung et al., 2021). In addition, the neuroprotective role of ILC2 cells was observed in the context of spinal cord injury (Gadani et al., 2017), after traumatic brain injury (TBI), during the early stage of stroke (Zheng et al., 2023), following intracerebral hemorrhage (Liu et al., 2023), and in neuromyelitis optica spectrum disorder, a severe CNS autoimmune disease that primarily damages the optic nerves and spinal cord (Kong et al., 2021). Upon CNS injury, meningeal ILC2s become activated in an IL-33-dependent manner and produce IL-13 both in the meninges and at the injury site where they are recruited. Although the functional impact of meningeal ILC2s on recovery from CNS injury was not determined, the adoptive transfer of lung-derived ILC2s has a beneficial effect on functional recovery (Gadani et al., 2017). In response to TBI, increased proliferation of ILC1, ILC2 and ILC3 subsets was observed within human meninges and CSF, and in murine meninges, where this effect lasted for up to 1 year after experimental TBI (Baban et al., 2021). An energy-sensing serine/threonine kinase, AMPK, regulates the expansion of meningeal ILCs in this case, including IL-33-mediated expansion of ILC2s. Administration of metformin, which activates AMPK, increased the frequency of ILC2s, which was associated with improved neurological outcomes, pointing to the beneficial role of ILC2s (Baban et al., 2021). In contrast to the protective role of ILC2s in aged mice and after CNS injury, ILC2s contribute to CNS demyelination in a mouse model of MS (Hirose et al., 2020). In this study, CNS demyelination was induced by ocular infection with HSV-IL-2, a recombinant herpes simplex virus 1 (HSV-1) that constitutively expresses mouse IL-2, a cytokine that is involved in demyelination during MS progression (Hirose et al., 2020). Demyelination was detected in the brain and spinal cord of ILC1^–/–^ and ILC3^–/–^ mice but not in ILC2^–/–^ mice, and adoptive transfer of ILC2s caused demyelination in the brain and spinal cord of ILC2^–/–^ recipient mice indicating that group 2 ILCs mediate CNS pathology induced by HSV-IL-2 (Hirose et al., 2020).

### Group 3 ILCs

Group 3 ILCs in the CNS were investigated in the context of EAE. ILC3 population is increased in circulation and the CNS of mice after induction of EAE (Grigg et al., 2021). ILC3 accumulation in the CNS during EAE is largely due to cell recruitment and not due to local proliferation (Hatfield and Brown, 2015). Accordingly, RNA sequencing analysis of sorted ILC3s in the CNS revealed that ILC3 transcriptionally expressed trafficking receptors *Ccr5*, *Itgal*, *Itgb2*, and *Itgb7* that are needed for the entry into the inflamed CNS (Grigg et al., 2021). ILC3 deficiency in mice with EAE reduced T-cell trafficking to the meninges (Hatfield and Brown, 2015), demonstrating an important role of ILC3s in T-cell maintenance within the CNS. Upon EAE induction, ILC3s in the CNS upregulate MHC-II and co-stimulatory molecules CD80 and CD86 (Grigg et al., 2021). In contrast, ILC3s in the blood of mice and humans do not express MHC-II, CD80, and CD86. ILC3s that express MHC-II (HLA-DR) and CD86 are also detected in the CSF of patients with MS (Grigg et al., 2021). Expression of these molecules by ILC3 is functionally important, as demonstrated by co-culture experiments showing that ILC3s sorted from the CNS during EAE promote antigen- and MHC-II-dependent production of the pro-inflammatory cytokines IFN-γ, TNF-α, IL-17A and granulocyte-macrophage colony-stimulating factor (GM-CSF) by myelin-specific CD4^+^ T-cells. The importance of ILC3s as antigen-presenting cells in the CNS parenchyma is also shown by the use of mice that lack MHC-II on ILC3s. Mice that lack MHC-II on ILC3s (*H2-Ab1*-floxed × Rorc^cre^) had significantly reduced numbers of IFN-γ, IL-17A and TNF-α-producing myelin-specific CD4^+^ T-cells in the CNS, and did not develop demyelinating disease (Grigg et al., 2021). Thus, antigen-presenting ILC3s promote pathological CD4^+^ T-cell responses in the CNS during autoimmune neuroinflammation (Grigg et al., 2021).

## Conclusion and perspectives

This article provides an overview of the involvement and function of ILCs within the CNS during physiological conditions and in the brain disorders. Even though ILCs are a minor population in healthy CNS and their functions overlap with those of T-cells, they can play an important role in CNS homeostasis and the development of CNS pathologies. ILCs can promote pathological CD4^+^ T-cell responses in the CNS during autoimmune neuroinflammation (Grigg et al., 2021), pathogenesis of ischemia (Gan et al., 2014; Zhang et al., 2014) and neurodegenerative diseases such as AD (Zhang et al., 2020) and ALS (Garofalo et al., 2020), and neurodevelopmental delay during CMV infection (Kveštak et al., 2021), but can also confer tissue protection (Gadani et al., 2017; Earls et al., 2020; Fung et al., 2020; Wang et al., 2023). Understanding ILC development and functions, as well as characterization of ILC subsets is continuously evolving. Thus, a better understanding of basic ILC biology in the context of neuroinflammatory conditions could explain some of the opposing findings regarding the involvement of ILCs in CNS disorders. Recent advances in the understanding of the acquisition of adaptive features by ILCs (Klose and Artis, 2020), raise a possibility that some of the ILCs could form adaptive populations of cells with specialized functions in CNS. Considering the importance of ILCs in CNS homeostasis and neuropathology, investigating origin and maintenance of these cells in the CNS and their interactions with other immune and CNS resident cells is of prime interest. Finally, a mechanistic understanding of how ILCs specifically act and respond to damage within the CNS leading to protective or pathological immune responses could be used to guide therapeutic interventions.

## Author contributions

DK: Conceptualization, Writing−original draft. AM: Writing−original draft. SJ: Writing−original draft, Conceptualization, Funding acquisition. IB: Conceptualization, Funding acquisition, Writing−original draft.
